The article "Study on the Effect of Sample Temperature on the Uniaxial Compressive Mechanical Properties of the Brain Tissue" was published in 2021. Journal: Appl Bionics Biomech.

# Study on the Effect of Sample Temperature on the Uniaxial Compressive Mechanical Properties of the Brain Tissue

**DOI:** 10.1155/2021/9986395

**Published:** 2021-07-14

**Authors:** Fengjiao Guan, Guanjun Zhang, Xiaohang Jia, Xiaopeng Deng

**Affiliations:** ^1^Laboratory of Science and Technology on Integrated Logistics Support, College of Intelligence Science and Technology, National University of Defense Technology, Changsha 410073, China; ^2^State Key Laboratory of Advanced Design and Manufacturing for Vehicle Body, Hunan University, Changsha 410082, China

## Abstract

Craniocerebral injury has been a research focus in the field of injury biomechanics. Although experimental endeavors have made certain progress in characterizing the material behavior of the brain, the temperature dependency of brain mechanics appears to be inconclusive thus far. To partially address this knowledge gap, the current study measured the brain material behavior via unconstrained uniaxial compression tests under low strain rate (0.0083 s^−1^) and high strain rate (0.83 s^−1^) at four different sample temperatures (13°C, 20°C, 27°C, and 37°C). Each group has 9~12 samples. One-way analysis of variance method was used to study the influence of sample temperature on engineering stress. The results show that the effect of sample temperature on the mechanical properties of brain tissue is significant under the high strain rate, especially at low temperature (13°C), in which the hardening of the brain tissue is very obvious. At the low strain rate, no temperature dependency of brain mechanics is noted. Therefore, the current results highlight that the temperature of the brain sample should be ensured to be in accordance with the living subject when studying the biomechanical response of living tissue.

## 1. Introduction

Craniocerebral injury is one of the common injuries and major causes of death in traffic accidents [1]. Marion showed that 84.1% of cases of severe craniocerebral trauma in children were caused by road traffic accidents and 72.5% of cases of severe craniocerebral trauma in adults were also caused by traffic accidents [2]. Therefore, craniocerebral injury has been a research hotspot in the field of injury biomechanics [1, 3–5]. Compared to biomechanical experiments that can be either hardly possible to perform due to moral reasons or extremely difficult associated with technical challenges and enormous expenses [6–12], the finite element simulation method is a particularly instrumental approach to evaluate the mechanical response of biological tissues under various load conditions and further uncover the mechanism of craniocerebral injury [4, 13, 14]. However, the biofidelity of the finite element model relies on accurate material constitutive parameters. Therefore, it is of great significance to study the factors affecting the constitutive parameters of brain tissue materials.

The article "Study on the Effect of Sample Temperature on the Uniaxial Compressive Mechanical Properties of the Brain Tissue" was published in 2021. Journal: Appl Bionics Biomech.

Brain tissue contains 70% water, 10%~12% lipids, 8% proteins, inorganic salts, organics, and carbohydrates [15]. Its high water content makes the volume modulus of the brain tissue almost equal to that of water with low shear resistance; the brain tissue is prone to shear deformation with respect to volume alteration [16, 17]. Thus far, the biomechanical properties of brain tissue were studied under various loading modes, such as stretching [11, 18, 19], compressing [10, 18, 20, 21], shearing [12, 18], and indentation method [5, 7]. The research indicated that the brain tissue is a medium exhibiting hyperelasticity [7, 10, 11, 19, 20, 22, 23], nonlinear elasticity [3], and nonlinear viscoelasticity [12, 18, 21]. These experimental data can be fitted by the constitutive models, through which the stresses are related to the strains in the form of mathematical expressions governed by model-specific material parameters. For example, Budday et al. compared the five commonly used constitutive models (e.g., neo-Hookean, Mooney Rivlin, Demiray, Gent, and Ogden) and pointed out that the Ogden model could better represent the hyperelasticity of brain tissue under stretching, compression, and shear conditions [12].

It should be pointed out that there are many factors affecting the mechanical properties of brain tissue, such as anatomical location [12, 13, 18], loading direction [1, 3, 13, 18], sample age [12, 13, 21], and temperature [1, 3, 4, 9, 20]. The experimental results obtained by different research teams are quite different. The mechanical heterogeneity of brain tissue and the inconsistency of test conditions are important reasons for the different experimental results. Although temperature has been recognized as one of the important factors affecting the mechanical properties of brain tissue [1, 3, 4, 20], consistent findings have not been reached yet. For example, Zambra et al. conducted the uniaxial compression test on fresh porcine brain tissue (coronal, *Ф*13 mm × 2 mm) using split-Hopkinson bar. The results showed that, when the strain was 10%, engineering stress and tangent modulus at storage temperature of 37°C are 3.5 times and 3.2 times than that of 0°C, respectively. By increasing the strain to 70%, engineering stress and tangent modulus at storage temperature of 37°C are 2.4 times and 2.2 times than that of 0°C, respectively [9]. Hrapko et al. studied the shear mechanical properties of fresh porcine brain tissue (corona radiata, *Ф*12 mm × 2 mm) at five temperatures of 37°C, 30°C, 23°C, 15°C, and 7°C (not explicitly stated as sample temperature or ambient temperature) and suggested that the dynamic shear modulus of brain tissue samples has a significant temperature dependence and the hardening phenomenon increases with decreasing temperature [1, 3]. Contrarily, Rashid et al. showed that there is no significant difference in unconstrained compression engineering stress of fresh porcine brain tissue samples (coronal, *Ф*15.0 mm × 6.1 mm) within the temperature range of 22°C to 37°C [20].

The article "Study on the Effect of Sample Temperature on the Uniaxial Compressive Mechanical Properties of the Brain Tissue" was published in 2021. Journal: Appl Bionics Biomech.

The above studies about the effect of temperature on the mechanical properties of brain tissue have reached inconsistent conclusions. This may be partially related to test methods and biomechanical response parameters. The above-mentioned study on the effect of temperature on the mechanical properties of brain tissue involves the sample preservation temperature, the test environment temperature, and the sample temperature. It is well known that longer preservation time affects the biomechanical properties of brain tissue [9, 24–26], so more fresh samples are used for biomechanical research. The ambient temperature will affect the temperature of the sample, which depends on the temperature difference between the two, the size of the sample, and the placing time, while the temperature of the sample itself is the direct factor affecting its mechanical properties. Therefore, this paper will study the influence of sample temperatures (13°C, 20°C, 27°C, and 37°C) on the mechanical properties of brain tissue under an unconstrained uniaxial compression test by controlling the consistency of sample temperature and ambient temperature.

## 2. Method

### 2.1. Sample Preparation

Twenty-four adult (about 8 months) fresh porcine brain tissue was obtained from the slaughterhouse and stored in a physiological saline solution at 4°C. The brain tissue was divided into two symmetrical hemispheres along the corpus callosum with a scalpel blade, and then the hemispheres were cut into slices about 6 mm thick using a combination cutter. With a cylindrical blade cutter (the inner diameter of the cutter is 9 mm) facing the section (coronal plane), a cylindrical sample with a diameter of about 9 mm and a height of about 6 mm mixed with gray matter and white matter was cut from the front to the back (as shown in Figure 1) [9, 20]. Two samples were prepared for each brain hemisphere and randomly assigned to low and high-speed compression tests. During the cutting process, 0.9% saline was continuously sprayed, and all the samples were tested within 6 hours in vitro.

### 2.2. Experimental Protocol

The experimental equipment is as shown in Figure 2. The air conditioning system was turned on to maintain the ambient temperature in the laboratory at the temperature required to carry out the test (13°C, 20°C, 27°C, and 37°C). The sample, together with the support plate, was placed on an INSTRON 5985 (Instron Corp., Norwood, MA USA) test machine. The sample was subjected to preheating treatment at a set temperature for about 2 minutes using an environmental chamber (MTS-651, Eden Prairie, MN USA), and the compression test was performed after the temperature of the sample reached the ambient temperature. Preheated phosphate-buffered saline (PBS) was sprayed on the support plate and press plate for lubrication to reduce the effect of friction on the biomechanical response of the sample [20]. The sample was preloaded at 0.02 N before formal loading [19, 27]. The compression speed was divided into low speed (0.05 mm/s) and high speed (5 mm/s). The corresponding strain rates were 0.0083 s^−1^ and 0.83 s^−1^, respectively. The compression ratio was controlled to 50% per compression test. Compression force in the experiment was measured by a force sensor (wmc-1000, Interface Inc., USA) with a range of 9.8 N and recorded by a data acquisition system (DT9838, Data Translation, USA) with a sampling frequency of 1000 Hz.

The article "Study on the Effect of Sample Temperature on the Uniaxial Compressive Mechanical Properties of the Brain Tissue" was published in 2021. Journal: Appl Bionics Biomech.

## 3. Results

Compression tests at four different sample temperatures (13°C, 20°C, 27°C, and 37°C) under two different loading rates (0.05 mm/s and 5 mm/s) were performed, and each sample was compressed to a strain of 50%. The ratio of the compressive force to the reference cross-sectional area of the specimen was defined as the engineering stress [20, 28]. Once the compression test was completed, all data were processed using Origin software to obtain the engineering stress-strain curves at two strain rates and specific temperatures, and the average engineering stress-strain curve and standard deviation curve were calculated using linear interpolation method [29, 30], as shown in Figures 3 and 4. The average engineering stress-strain curves corresponding to the temperatures of the four samples under two different strain rates are shown in Figure 5. Under the condition of low strain rate, the influence of sample temperature on the engineering stress-strain curve was not obvious. Under high strain rate conditions, the engineering stress-strain curves at 20°C, 27°C, and 37°C were not significantly different, and the engineering stress at 13°C was significantly higher than those of the other three samples.

In order to study the influence of sample temperature on the mechanical properties of the sample, the corresponding engineering stress of samples was analyzed when the strain was 50%. The results are shown in Table 1. When the strain rate was 0.0083 s^−1^, the engineering stresses were 2.45 ± 0.82 kPa, 2.39 ± 0.40 kPa, 2.24 ± 0.77 kPa, and 2.09 ± 0.56 kPa at 13°C, 20°C, 27°C, and 37°C, respectively. At a strain rate of 0.83 s^−1^, the engineering stresses under a strain of 0.5 were 5.85 ± 1.90 kPa at 13°C, 3.37 ± 0.43 kPa at 20°C, 3.10 ± 0.90 kPa at 27°C, and 3.19 ± 1.16 kPa at 37°C.

The article "Study on the Effect of Sample Temperature on the Uniaxial Compressive Mechanical Properties of the Brain Tissue" was published in 2021. Journal: Appl Bionics Biomech.

The effects of temperature on engineering stress at two strain rates were investigated using one-way ANOVA. Under low-speed compression conditions, the effect of temperature on engineering stress was not significant (*p* = 0.576). However, under high-speed compression conditions, the temperature had a significant effect on engineering stress (*p* < 0.001). The difference of engineering stress between samples at different temperatures was further studied by using multiple comparison between groups, as shown in Figure 6. At low strain rate (0.0083 s^−1^), the engineering stress gradually decreased with the increase of temperature, but the difference between the groups was not statistically significant (*p* > 0.05). At high strain rate (0.83 s^−1^), the engineering stress of the specimen at 13°C is significantly different from that of the specimen at 20°C (*p* = 0.001), 27°C (*p* < 0.001), and 37°C (*p* < 0.001), and there was no statistically significant difference in engineering stress between samples at 20°C, 27°C, and 37°C (*p* > 0.05).

## 4. Discussion

In this paper, the uncompressed uniaxial compression tests at different loading rates (0.05 mm/s and 5 mm/s) were used to study the compression mechanical properties of brain tissue at different sample temperatures (13°C, 20°C, 27°C, and 37°C). The effect of sample temperature on the compression performance of brain tissue under high strain rate conditions was obvious, especially when the sample temperature was 13°C, the hardening phenomenon of brain tissue was obvious (as shown in Figure 5). One-way ANOVA also showed that the temperature of the sample had a significant effect on the engineering stress at high strain rate (*p* < 0.001). Therefore, the temperature of brain tissue samples should be consistent with the in vivo state in the study aimed at exploring the biomechanical test of living tissue.

The results of this study also showed that there is no significant difference in the engineering stress of brain tissue at the sample temperature of 20-37°C regardless of low strain rate (0.0083 s^−1^) and high strain rate (0.83 s^−1^) (*p* = 0.727~0.961). Rashid et al. also carried out an unconstrained uniaxial compression test of brain tissue at dynamics train rates of 30 and 50 s^−1^ at 22°C and 37°C and pointed out that at 22°C and 37°C, there is no statistically significant difference in the engineering stress of brain tissue (*p* = 0.856~0.929). In this study, between 20°C and 37°C, a group of 27°C brain samples was added, and the loading rate extends to quasistatic, which further illustrated that there is no significant difference in the engineering stress of brain tissue within the sample temperature range of 20~37°C. This is consistent with the results of Rashid et al. [20]. Therefore, the mechanical properties of brain tissue obtained from experiments conducted at room temperature in the literature can still be used with caution.

The article "Study on the Effect of Sample Temperature on the Uniaxial Compressive Mechanical Properties of the Brain Tissue" was published in 2021. Journal: Appl Bionics Biomech.

Hrapko et al. analyzed the shear mechanical properties of fresh porcine brain samples at different temperatures of 37°C, 30°C, 23°C, 15°C, and 7°C at a strain rate of 1 s^−1^. The results showed that the dynamic shear modulus of brain tissue was obviously temperature-dependent and the hardening response increased obviously with the decrease of temperature [1, 3]. In this study, when the sample temperature was 13°C, the engineering stress increased significantly (*p* = 0.000) with the decrease of temperature under the condition of high strain rate, which was consistent with the results obtained by Hrapko et al.

The experimental results in this study also showed that the sample temperature had no significant effect on the compression response of brain tissue at low strain rate, but it had a significant effect at high strain rate. Therefore, the strain rate may also play a role in the effect of sample temperature on the mechanical properties of brain tissue, and it is necessary to further study it in the future.

In this study, the engineering stress of brain tissue was used to analyze the influence of sample temperature. In the finite element model, the biomechanical properties of brain tissue can be characterized by various material constitutive models and corresponding parameters. Therefore, it is more meaningful to explore the influence of temperature on the constitutive parameters of materials in the future.

## 5. Conclusion

Because the sample temperature is affected by the ambient temperature, it is more valuable to explore the mechanical properties of the brain tissue at the sample temperature. In this study, 81 samples were prepared from 24 porcine brains and randomly divided into 8 groups. The effects of sample temperature (13°C, 20°C, 27°C, and 37°C) on the uniaxial compression mechanical properties of the brain tissue under low (0.05 mm/s) and high (5 mm/s) loading rates were studied, respectively. With the decrease of the temperature of the sample, the engineering stress of the brain tissue was gradually increased. The results of one-way ANOVA showed that the effect of sample temperature on the mechanical properties of brain tissue was not statistically significant (*p* = 0.576) at low strain rate. At high strain rates, the influence of sample temperature on the mechanical properties of brain tissue is significant (*p* < 0.001). When the sample temperature is in the range of 27-37°C, the difference in the biomechanical response of the brain tissue is not obvious. When the sample temperature is lower than 14°C, the brain tissue at high strain rates appears obvious hardening. Therefore, it is necessary to control the sample temperature during the brain tissue test to obtain accurate brain tissue biomechanical response, especially under high strain rate conditions.

The article "Study on the Effect of Sample Temperature on the Uniaxial Compressive Mechanical Properties of the Brain Tissue" was published in 2021. Journal: Appl Bionics Biomech.

## Figures and Tables

**Figure 1:** Preparation of brain tissue specimen.

**Figure 2:** The setup of brain tissue compression test.

**Figure 3:** The compression engineering stress-strain curves of brain tissue under low strain rate (0.0083 s^−1^) condition. (a) 13°C; (b) 20°C; (c) 27°C; (d) 37°C.

**Figure 4:** The compression engineering stress-strain curves of brain tissue under high strain rate (0.83 s^−1^) condition. (a) 13°C; (b) 20°C; (c)27°C; (d) 37°C.

**Figure 5:** The average engineering stress-strain curves of brain tissue at different temperatures. (a) Low strain rate 0.0083 s^−1^; (b) high strain rate 0.83 s^−1^.

**Figure 6:** The specimen engineering stress at 50% engineering strain and inter group multiple comparison at four different temperatures. (a) Low strain rate 0.0083 s^−1^; (b) high strain rate 0.83 s^−1^.

**Table 1:** The maximum engineering stress of sample under different conditions.

Strain rate (s^−1^)	Temperatures (°C)	Engineering strain (kPa)	Sample size
0.0083	13	2.45 ± 0.82	10
	20	2.39 ± 0.40	10
	27	2.24 ± 0.77	9
	37	2.09 ± 0.56	11

0.83	13	5.85 ± 1.90	12
	20	3.37 ± 0.43	9
	27	3.10 ± 0.90	9
	37	3.19 ± 1.16	11

## Data Availability

The data used to support the findings of this study have not been made available because the data also forms part of an ongoing study.
